# Rhodiola Rosea Extract Counteracts Stress in an Adaptogenic Response Curve Manner via Elimination of ROS and Induction of Neurite Outgrowth

This article has been retracted.

**DOI:** 10.1155/2022/5647599

**Published:** 2022-05-13

**Authors:** Anastasia Agapouda, Amandine Grimm, Imane Lejri, Anne Eckert

**Affiliations:** ^1^University of Basel, Transfaculty Research Platform, Molecular and Cognitive Neuroscience, Neurobiology Lab for Brain Aging and Mental Health, Basel, Switzerland; ^2^Psychiatric University Clinics, Basel, Switzerland

## Abstract

**Background:**

Sustained stress with the overproduction of corticosteroids has been shown to increase reactive oxygen species (ROS) leading to an oxidative stress state. Mitochondria are the main generators of ROS and are directly and detrimentally affected by their overproduction. Neurons depend almost solely on ATP produced by mitochondria in order to satisfy their energy needs and to form synapses, while stress has been proven to alter synaptic plasticity. Emerging evidence underpins that *Rhodiola rosea*, an adaptogenic plant rich in polyphenols, exerts antioxidant, antistress, and neuroprotective effects.

**Methods:**

In this study, the effect of *Rhodiola rosea* extract (RRE) WS®1375 on neuronal ROS regulation, bioenergetics, and neurite outgrowth, as well as its potential modulatory effect on the brain derived neurotrophic factor (BDNF) pathway, was evaluated in the human neuroblastoma SH-SY5Y and the murine hippocampal HT22 cell lines. Stress was induced using the corticosteroid dexamethasone.

**Results:**

RRE increased bioenergetics as well as cell viability and scavenged ROS with a similar efficacy in both cells lines and counteracted the respective corticosteroid-induced dysregulation. The effect of RRE, both under dexamethasone-stress and under normal conditions, resulted in biphasic U-shape and inverted U-shape dose response curves, a characteristic feature of adaptogenic plant extracts. Additionally, RRE treatment promoted neurite outgrowth and induced an increase in BDNF levels.

**Conclusion:**

These findings indicate that RRE may constitute a candidate for the prevention of stress-induced pathophysiological processes as well as oxidative stress. Therefore, it could be employed against stress-associated mental disorders potentially leading to the development of a condition-specific supplementation.

## 1. Introduction

*Rhodiola rosea* is a perennial flowering plant belonging to the Crassulaceae family. It grows naturally in the wild at high altitude and can be found in the Arctic and in mountainous areas of Central Asia and Europe [1]. Extracts from *Rhodiola* are considered as adaptogens (EMEA/HMPC/102655/2007). Adaptogens are nontoxic agents that increase resistance against physical, chemical, biological, and psychological stressors by normalizing the harmful effect of these stressors independently of the nature of the pathologic state. In this way, they help the organism to achieve a physiological equilibrium and homeostasis during stressful situations [2, 3]. Historically, *Rhodiola rosea* had been used by Vikings to increase their endurance and physical strength [4]. Clinical studies have indicated beneficial effects of *Rhodiola rosea* extracts (including the WS®1375 extract) in stress and fatigue management as well as in building resilience [5–13]. RRE has also shown antioxidant, anti-inflammatory, and neuroprotective effects in animal [14–17] and cellular models [18]. Phytochemically, extracts of *Rhodiola rosea* roots and rhizomes contain mainly six classes of compounds: flavonoids, phenolic acids, phenylethanoloids, phenylpropanoids, monoterpenes, and triterpenes. Salidroside, a phenylethanol glycoside, is considered as the main pharmacologically active compound of *Rhodiola rosea*, although it is also found in many other *Rhodiola* species. On the contrary, some cinnamic alcohol glycosides such as rosavin, rosarin, and rosin have been solely found in *Rhodiola rosea*. These compounds are referred to as “rosavins” and are represented by the phenylpropanoid rosavin [1]. Both salidroside and rosavin represent the lead marker compounds of the RRE. Extracts of *Rhodiola rosea* rhizomes and roots have been characterized as “traditional herbal medicinal product for temporary relief of symptoms of stress, such as fatigue and sensation of weakness” by the European Medicines Agency (EMA) (EMEA/HMPC/102655/2007). Although there is already published research on the individual RRE compound markers [19–22], limited studies have examined cellular and molecular mechanisms underlying the action of the whole RRE using in depth in vitro methods.

Stress is defined as a state of threatened or recognized as threatened homeostasis. In response to this threatened situation, organisms are armed with a highly sophisticated system, namely, the stress system which supplies the organisms with the proper central and peripheral neuroendocrine adaptive responses. Although the stress response is crucial for survival and adaptation, excessive, insufficient, or prolonged responses might be harmful for physiological functions, including metabolism, growth, circulation, and immune responses as well as reproduction to name a few [23]. The main elements of the stress system are the hypothalamic-pituitary-adrenal (HPA) axis and the sympathetic nervous system. The HPA axis consists of the hypothalamus, the pituitary gland, and the adrenal cortex. Acute activation of the HPA axis upon stressful events, the so-called eustress, increases the overall functions of the organism [24, 25]. However, sustained activation over a long period of time exerts detrimental effects as overaccumulation of glucocorticoids becomes deleterious for the brain but also for other systems in the body, a phenomenon called allostatic load [23, 26]. It has been shown that glucocorticoids regulate mitochondrial, neuronal, and synaptic functions in an inverted “U-shape” manner in which low to moderate levels of stress increase the overall functions, while intense or sustained stress exhibits harmful effects. [24, 25, 27, 28]. Indeed, treatment of primary cortical neurons with both low and high corticosterone concentrations increased mitochondrial membrane potential (MMP), calcium holding capacity, and neuronal survival after a short-term treatment of 1.5 hours showing a neuroprotective effect. However, treatment of the same cells with high concentrations over a long-term treatment of 3 days decreased all the aforementioned functions and had a detrimental effect on neurons [28]. Neurons rely on mitochondria to satisfy their energy requirements and to accomplish their functions including synaptic plasticity. Neuronal mitochondria are constantly transported through microtubule networks where metabolic and energy needs rise [29, 30]. Most of the brain energy is invested at synapses in order to preserve ion gradients and enable the signaling processes of neurotransmission. It seems that glucocorticoids exert effects via a convergent mitochondrial, neuronal, and synaptic pathway [29]. While GR (glucocorticoid receptor) signaling is crucial for glucocorticoid-affected mitochondrial function and spine plasticity, brain-derived neurotrophic factor (BDNF) signaling plays a major role for synaptic plasticity and mitochondrial function [31–33]. BDNF acts via its receptor TrkB and can influence GR-mediated gene expression [34]. BDNF signaling promotes the phosphorylation of GR at serines 134 and 267 through activation of the cofactor CREB1 (CAMP responsive element binding protein 1) to induce a new gene expression signature. Interestingly, stress-related disorders are often characterized by increased levels of circulating cortisol and reduced BDNF levels [35]. Moreover, glucocorticoid stress has been shown to increase oxidative stress upon binding of glucocorticoids to GRs [28].

In this in vitro study, we first aimed to evaluate the effect of the RRE WS®1375 on neuronal bioenergetics and neurite outgrowth, as well as its potential modulatory effect on the BDNF pathway. Then, we evaluated the potency of the RRE WS®1375 to neutralize glucocorticoid stress-induced ROS generation and to prevent the stress-related decrease in cell viability and neurite outgrowth.

## 2. Materials and Methods

### 2.1. Chemicals and Reagents

Dulbecco's-modified Eagle medium (DMEM), phosphate-buffered saline (PBS), fetal calf serum (FCS), Hanks' Balanced Salt solution (HBSS), penicillin/streptomycin, dihy-drorhodamine 123 (DHR), 2',7'-dichlorodihydrofluorescein diacetate (DCF), thiazolyl blue tetrazolium bromide (MTT), neurobasal medium, retinoic acid, paraformaldehyde, bovine serum albumin (BSA), 4′,6-Diamidino-2-phenylindol (DAPI), Triton X-100, and dexame-thasone were purchased from Sigma-Aldrich (St. Louis, MO, USA). Alexa Fluor 488 and *β*III-tubulin antibodies were from R&D Systems (MN, USA). MitoSOX, glutaMax, and B27 supplement were from Gibco Invitrogen (Waltham, MA, USA). NGF was from Lubio (Zürich, Switzerland), ATPlite1step kit from PerkinElmer (Waltham, MA, USA) and horse serum (HS) from Amimed, Bioconcept (Allschwil, Switzerland). Recombinant human BDNF protein was from Novus Biologicals (Littleton, CO, USA). The mature BDNF rapid ELISA kit from Biosensis (Adelaide, Australia), the RNA extraction kit from Qiagen (Hilden, Germany), the GoScript™ Reverse Transcription Mix, Oligo, and the GoTaq® Master Mix for real-time quantitative PCR (RT-qPCR) from Promega (Dübendorf, Switzerland) were purchased. The primers for BDNF (Fw: 5′-AAG CAA TAC TTC TAC GAG ACC AA-3′; Rev: 5′-CTT ATG AAT CGC CAG CCA ATT-3′), TrkB (Fw: 5′-CCG AGA TTG GAG CCT AAC AG-3′; Rev: 5′-CAC CAG GAT CAG TTC AGA CAA-3′), p75NTR (Fw: 5′-GCC TTC AAG AGG TGG AAC A-3′; Rev: 5′-CGC AGA GCC GTT GAG AAG-3′), and the housekeeping gene GAPDH (Fw: 5′-CAA GGT CAT CCA TGA CAA CTT TG-3′; Rev: 5′-GGG CCA TCC ACA GTC TTC TG-3′) were from Microsynth (Balgach, Switzerland).

### 2.2. Characterization of RRE WS®1375

WS®1375, a proprietary dry extract from *Rhodiola rosea* roots and rhizomes harvested in Russia, was supplied by Dr. Willmar Schwabe GmbH & Co. KG (Karlsruhe, Germany). WS®13751 was obtained by extraction with 60% (w/w) aqueous ethanol (drug extract ratio 1.5-5 : 1). The quantification of rosavins (assessed as rosavin) and salidroside (assessed as p-tyrosol) in WS®1375 was conducted by reversed-phase high-performance liquid chromatography (HPLC) with UV detection. For quantification of salidroside, p-tyrosol was used for calibration of the peak area. After the integration of the salidroside peak, the value was multiplied with the factor of 2.173 to correct the amount according to the molecular mass difference between salidroside/p-tyrosol (300.31/138.16 = 2.173). The HPLC-UV chromatograms were recorded on Merck HPLC equipment using a Merck LiChrospher® 100 C18 (5 *μ*M, 4 × 250 mm) column with precolumn conditioning at 25°C. Eluent A consisted of demineralized water with 0.3% (v/v) o-phosphoric acid 85%. Eluent B consisted of acetonitrile. At a flow rate of 1 ml/min, the gradient was as follows: from 0.0 to 30.0 min; linear from 5% to 20% eluent B, from 30.0 to 45.0 min; linear from 20% to 50% eluent B, from 45.0 to 45.5 min; linear from 50% to 5% eluent B, from 45.5 to 60.0 min; and isocratic 5% eluent B as equilibration period, resulting in a total run time of 60.0 min. UV detection wavelength was 251 nm for rosavins and 275 nm for salidroside, and a column temperature of 25°C was applied. The injection volume was 10 *μ*l of a 4 mg/ml RRE WS®1375 dissolved in methanol. Calculations were conducted using the software EZChrom. Visualization of the chromatogram was done with ACD/Labs Spectrus Processor (v2017.2.1) software.

### 2.3. Cell Culture

The human neuroblastoma SH-SY5Y cell line (ATCC® CRL-2266™ Manassas, VA, USA) was selected as our cellular model in this study as it is a well-established and widely used neuronal model in biochemical studies in general as it expresses neuronal receptors. In parallel, the murine hippocampal cell line HT22 (SCC129, Sigma-Aldrich, St. Louis, MO, USA) was used for confirmation of results and because the hippocampus is directly affected by corticosteroid stress. The SH-SY5Y cells were kept and grown at 37°C in a humidified incubator chamber under an atmosphere of 5% CO_2_ in DMEM supplemented with 10% (v/v) heat-inactivated FCS, 5% HS, 2 mM glutaMax, and 1% (v/v) penicillin/streptomycin. The HT22 cells were cultured in DMEM containing 10% FCS, 1% penicillin-streptomycin, and 1% glutaMax. Cells were passaged 1-2 times per week, and the cells used for the experiments did not exceed passage 20. The cells were plated when they reached 80–90% confluence.

To study the neurite outgrowth on differentiated SH-SY5Y cells, cell plates were coated with collagen type I (Rat tail, Corning, Amsterdam, Netherlands) at 0.05 mg/ml.

### 2.4. Treatment of Cells

Evaluation of cell viability (MTT assay) was conducted on SH-SY5Y and HT22 cells to determine the potential toxic concentration range of the WS®1375 RRE. Initially, the RRE was screened in a broad concentration range from 1 ng/ml to 500 ng/ml (see Suppl. Tables 1 and 2). Stock solution of the RRE was prepared in DMSO (final assay concentration of DMSO <0.0001%, which is the concentration of DMSO present in 500 ng/ml RRE). There was no effect of the vehicle solution alone (0.005% DMSO) compared to the untreated condition (see Suppl. Tables 1 and 2). Therefore, only the untreated control condition is presented in the results section. The first screening revealed that RRE did not show significant toxic effects on the neuroblastoma and hippocampal cells up to a concentration of 500 ng/ml. According to the results of the first screening, a concentration range from 1 ng/ml to 100 ng/ml was tested in a second screening cycle. The screening was conducted by using an ATP detection assay (ATPlite 1step kit was from PerkinElmer) and a cell viability assay (MTT assay).

For the experiments evaluating the effect of RRE per se, cells were plated and treated 1 day after plating for 24 h either with DMEM (untreated cells-control condition) or with a final concentration of 1 ng/ml to 100 ng/ml of the extract (namely, 1, 5, 10, and 100 ng/ml).

Dexamethasone (Dexa), an agonist of the glucocorticoid receptor, was used to induce stress on the SH-SY5Y and HT22 cells. Dexa mimics the effect of the stress hormone cortisol as they are both binding at the same receptors. Dexa was dissolved in DMSO, and then, subsequent working solutions were generated for the treatment of the cells. Dexa at 100 *μ*M was able to decrease the cell viability of HT22 cells. while the viability of SH-SY5Y cells was decreased after treatment with Dexa at 400 *μ*M. These Dexa concentrations were selected based on screening experiments conducted on SH-SY5Y and HT22 cells using the MTT reduction assay. For the ROS experiments, a much lower Dexa concentration could induce oxidative stress, namely, 5 *μ*M for HT22 cells and 100 *μ*M for SH-SY5Y cells.

For the stress experiments, two treatment strategies were tested: preventive and curative. First, cells were pretreated for 24 h with RRE (1, 5, 10, and 100 ng/ml) and then treated for another 24 h with the respective Dexa concentration (= preventive treatment). Or, cells were first pretreated for 3 h with Dexa and then treated for another 24 h with RRE (1, 5, 10, and 100 ng/ml = curative treatment). Each assay was conducted and repeated at least in triplicate.

### 2.5. ATP levels

Total ATP content was determined using a bioluminescence assay (ATPlite 1step) according to the instructions of the manufacturer and as previously described [36, 37]. SH-SY5Y and HT22 cells were plated in 6 replicates into white 96-well cell culture plates at a density of 1 × 10^4^ cells/well and 5 × 10^3^ cells/well, respectively. The ATP was extracted from the cells upon lysis, and it was transformed into light. The method measures the formation of light from ATP and luciferin catalyzed by the enzyme luciferase. The emitted light was linearly correlated to the ATP concentration and was measured using the multimode plate reader Cytation 3 (BioTek instruments, Winooski, VT, USA).

### 2.6. Cell Viability Assay

Cell viability was investigated using a MTT cell proliferation assay. After treatment, the cells were incubated with MTT (3-(4,5-dimethylthyazol-2-yl)-2,5-diphenyl-tetrazolium bromide) in DMEM for 3 hours. MTT is reduced to a violet formazan derivative by mitochondrial enzymatic activity. At the end of the reaction, the cells were dissolved in DMSO 100%. MTT absorbance was measured at 595 nm using the multimode plate reader Cytation 3.

### 2.7. Determination of ROS Levels

Mitochondrial and cytosolic ROS levels as well as the specific levels of mitochondrial superoxide anion radical levels were assessed using the fluorescent dyes dihydrorhodamine 123 (DHR), 2′,7′-dichlorodihydrofluorescein diacetate (DCF), and the red mitochondrial superoxide indicator (MitoSOX), respectively, as previously described ([37]; Schmitt, [38]). SH-SY5Y and HT22 cells were plated in 6 replicates into black 96-well cell culture plates at a density of 1 × 10^4^ cells/well and 5 × 10^3^ cells/well, respectively. After treatment, cells were incubated with 10 *μ*M of one of the dyes: DHR or DCF for 20 min or 5 *μ*M of MitoSOX for 90 min at room temperature in the dark on an orbital shaker. After washing the cells three times with HBSS, the formation of green fluorescent products triggered by DHR and DCF, respectively, was detected at 485 nm (excitation)/535 nm (emission). MitoSOX triggers the formation of red fluorescent products which were detected at 531 nm (excitation)/595 nm (emission). The intensity of fluorescence was proportional to mitochondrial ROS, cytosolic ROS, and mitochondrial superoxide anion levels. The fluorescence was measured using the Cytation 3 multimode plate reader.

### 2.8. Neurite Outgrowth Determination

SH-SY5Y neuroblastoma cells were plated in black 96-well plates that were precoated with collagen 0.05 mg/ml. 24-h postplating, cell differentiation was induced by adding neurobasal medium containing 2% B27 supplement, 1% penicillin-streptomycin, 1% glutaMax, and 10 *μ*M retinoic acid (RA) for 3 days as described previously [39]. To assess the effects of WS®1375 RRE in physiological condition, cells were treated either with the RRE at the concentrations 5 and 10 ng/ml. A treatment with 50 ng/ml of NGF or 50 ng/ml of BDNF was used as positive controls. To assess the effects of WS®1375 RRE under stress condition, cells were first treated with 100 *μ*M Dexa and then treated with 5 ng/ml RRE. After 3 days of treatment, cells were fixed with 2% paraformaldehyde.

### 2.9. Immunostaining

The usage of black 96-well plates with a clear bottom allows to directly image the samples. Immunolabeling of neurites was performed using an anti-*β*III-tubulin primary antibody and Alexa Fluor 488-conjugated secondary antibody (fluorescence emission in the green wavelength). Immunolabeling of the nucleus was conducted using DAPI (4′,6-diamidino-2-phenylindole) which emits blue fluorescence upon binding to adenine and thymine-rich regions of DNA.

### 2.10. Microscopy and Analysis (Software)

Images were taken using Cytation 3, a digital cell imaging multimode reader with a 20× objective. Analysis was performed using ImageJ (Neurophology plugin) software to evaluate parameters of neuroplasticity as described before [39]: neurite count, total neurite length, number of branching points = attachment point, and number of contact points = endpoint.

### 2.11. RNA Extraction and Quantitative Real-Time PCR

SH-SY5Y cells were plated at 6-well plates at a density of 4 × 10^5^ cells/well. To assess the effects of RRE on gene expression, the cells were treated 24-h postplating either with DMEM (control condition) or with WS®1375 RRE at 5 ng/ml. Cells were lysed after 1 h, 2 h, 3 h, 4 h, and 24 h of treatment. To investigate the effects of RRE on gene expression in stress condition, cells were treated with Dexa for 3 h and then treated with RRE (5 ng/ml). Based on the data obtained in physiological condition (without Dexa), cells were lysed after 24 h of RRE treatment.

Total RNA was isolated with RNeasy spin columns (Qiagen, Hilden, Germany). Quantitation was performed by spectrophotometry (Nanodrop, Thermoscientific). One microgram of RNA from each sample was subjected to reverse transcription using the GoScript™ Reverse Transcription Mix from Promega (Dübendorf, Switzerland). After reverse transcription the cDNA was diluted 1 : 5 with nuclease-free water, and each cDNA sample was amplified using quantitative real-time PCR (StepOne™ System, Applied Biosystems). Each PCR contained 900 nM of each primer (forward and reverse), the PCR MasterMix (GoTaq® qPCR Master Mix, Promega), and CXR reference dye combined in 17 *μ*l as well as 3 *μ*l of the diluted cDNA. 40 cycles were performed of the following thermal profile: 2 min at 95°C, 15 sec at 95°C followed by 1 min at 60°C. Final quantitation was conducted using the comparative CT method (threshold cycle: number of cycle until sample signal is detected). GAPDH was used as control housekeeping gene to assess the validity of the cDNA mixture and the PCR reaction.

### 2.12. Determination of Mature BDNF Protein Level

SH-SY5Y cells were plated in 10 cm^2^ dishes. 24-h postplating, the cells were treated either with DMEM (control condition) or with WS®1375 RRE at 5 ng/ml. Cell lysates were produced after 4 h and 24 h of treatment. The time points were selected according to published data on the detection of BDNF levels in rats and mice [22, 40, 41] as well as in neuronal cells [22, 41]. The concentrations of mature BDNF were quantified in duplicate using the Biosensis Mature BDNF Rapid ELISA Kit (Thebarton, Australia) according to the instructions of the manufacturer. Prior to each immunoassay, cell lysates were diluted 1 : 4 using the provided sample buffer. After incubation, the absorbance was measured at 450 nm using the Cytation 3 multimode plate reader, and the levels of mature BDNF were calculated in pg/ml and normalized to 1 mg of total protein level.

### 2.13. Statistical Analysis

Data are given as the mean ± SEM, normalized to the untreated control group (=100%). Statistical analyses were performed using the Graph Pad Prism software version 5.02. For statistical comparisons, one-way ANOVA was used, followed by Dunnett's multiple comparison tests versus the control or versus Dexa or Student *t* test. *p* values <0.05 were considered statistically significant. The adequacy of fits was estimated by the *R*-squared value (>0.9) using Pearson correlation and linear regression analysis.

## 3. Results

### 3.1. Characterization of the Lead Compounds of RRE WS®1375

The lead compounds in the RRE WS®1375 were determined by reversed-phase HPLC with UV detection (Figure 1). The single WS®1375 batch used for the present study contained 1.04% rosarin, 2.63% rosavin, 1.04% rosin (all assessed as rosavins), and 1.16% salidroside (assessed as p-tyrosol) that is in agreement with the concentration range of those lead compound in RREs used for medicinal purposes in other studies [42] .

### 3.2. RRE Increases Bioenergetics and Cell Metabolic Activity in SH-SY5Y and HT22 Cells

To examine the effect of the extract in physiological (healthy) condition, a screening was conducted using the ATP production assay and the cell viability (MTT) assay which is an indicator of increased mitochondrial metabolic activity. Regarding SH-SY5Y cells, all tested concentrations (1, 5, 10, and 100 ng/ml) significantly increased the ATP levels up to 8.3% (Figure 2(a)). The same effect was observed in the cell viability assay in which all the concentrations increased the MTT values up to 12.1%. The highest increase amounted to 12.1% and 11.5% and was caused by treatment with 5 and 10 ng/ml, respectively (Figure 2(b)). Upon Pearson correlation of the ATP production with the cell viability assay, a significant positive linear correlation was found in SH-SY5Y cells (*R*^2^ = 0.9007, *p* = 0.0137) with the most effective RRE concentrations being 5 and 10 ng/ml. The resulting plot allows clear visualization of the most effective concentrations of RRE (Figure 2(c)). This suggests that the improvement in ATP production was preferentially linked to an increase in metabolic activity of the cells. These results were confirmed in the HT22 cells in which the effects of RRE were like those observed in SH-SY5Y cells. In detail, all tested concentrations (1-100 ng/ml) increased both bioenergetics, in the form of ATP production, and metabolic activity, in the form of cell viability of up to 18.8% and 19.7%, respectively (Figures 2(d) and 2(e)). The RRE concentration with the most prominent effect was 5 ng/ml in both assays which is also apparent in the Pearson correlation plot in 2F. Again, a significant positive linear correlation was found between the ATP production and the cell survival assays in HT22 cells (*R*^2^ = 0.8616, *p* = 0.0228) (Figure 2(f)).

Overall, these data showed that RRE increases ATP production and cell metabolic activity in two different cell lines in an inverted U-shape manner, with 5 and 10 ng/ml being the most efficient extract concentrations.

### 3.3. RRE Promotes Neurite Outgrowth in Differentiated SH-SY5Y Cells

The capacity of RRE in promoting neurite outgrowth was assessed in differentiated SH-SY5Y cells [39]. The two most promising concentrations from the previous experiments, 5 and 10 ng/ml, were tested in the subsequent experiments on neurite outgrowth (Figure 3(a)). The neurotrophins nerve growth factor (NGF) and brain-derived neurotrophic factor (BDNF), both at 50 ng/ml, which are known inducers of neurite outgrowth and promoters of cell survival and synaptic plasticity, were used as positive controls. The cells were treated for three days. After immunostaining and microscopy analysis, we showed that RRE promoted a significant neurite outgrowth which was visually comparable to the effect caused by the positive controls (Figure 3(a)). To confirm and quantify the observed effects, the ImageJ (Neurophology plugin) software was used for analysis which allows the measurement of specific neurite outgrowth parameters such as neurite count, total neurite length, attachment points of neurons, and endpoints of neurons (Figures 3(b)–3(e)). The extract conditions as well as the positive controls were normalized and compared to the untreated control cells. As expected, the positive controls induced a considerable increase in all the parameters. Interestingly, treatment of the cells with the RRE at 5 and 10 ng/ml had a similar effect to the positive controls. Specifically, the concentrations 5 and 10 ng/ml caused an increase of 90.1% and 64.3%, respectively, in neurite count; an increase of 104% and 61.8%, respectively, in total neurite length; an increase of 101% and 67.8%, respectively, in the number of attachment points; and an increase of 98.7% and 61.6%, respectively, in the number of endpoints (Figures 3(b)–3(e)).

### 3.4. RRE Increases the BDNF mRNA Expression and the Mature BDNF Protein Level in SH-SY5Y Cells

Determination of the effect of the RRE on the BDNF gene expression was conducted via quantitative real-time PCR in SH-SY5Y cells. Cells were treated either with plain medium (DMEM) or with RRE 5 ng/ml, and cell lysates were collected 1 h, 2 h, 3 h, 4 h, and 24 h after treatment. RRE had an upregulating effect on BDNF gene expression (Figure 4(a)). The effect peaked after 3 h of treatment and decreased afterwards, but still exhibited a significant increase of mRNA expression levels after 4 h and 24 h of treatment.

Determination of the effect of RRE on the mature BDNF protein level was conducted via an enzyme immunoassay specifically detecting the mature form of BDNF protein. Cells were treated with either plain medium (DMEM) or RRE at a concentration of 5 ng/ml. Cell lysates were collected after 4 h and 24 h of treatment. Mature BDNF concentration is quantified and is illustrated in Figure 4(b). Treatment with RRE had a significantly upregulating effect on the protein level of mature BDNF at 4 h and 24 h, which is in line with the BDNF mRNA expression profile.

Together, these data indicate that RRE increases BDNF gene expression and protein level, which may be linked to the effects observed on neurite outgrowth.

### 3.5. RRE Eliminates ROS and Rescues Cell Metabolic Activity Caused by Dexamethasone

Glucocorticoid-related stress has been shown to induce oxidative damages in cells [27]. Therefore, in a next step, we aimed to assess whether RRE exerted protective effects in stress condition. Dexamethasone (Dexa), a synthetic agonist of the glucocorticoid receptor which mimics the effect of cortisol, was used to induce stress. The capacity of RRE to counteract the detrimental effects of glucocorticoid stress was examined in two treatment strategies: a preventive treatment in which SH-SY5Y cells where first treated with RRE for 24 h before to be exposed to stress (Dexa 100 *μ*M for 24 h), and a curative treatment in which SH-SY5Y cells were treated with Dexa 3 h before treating with RRE for an additional 24 h.

Dexa 100 *μ*M caused a significant elevation in cytosolic ROS, mitochondrial ROS, and mitochondrial superoxide anion levels, respectively, in SH-SY5Y cells (Figures 5(a)–5(C) and 5(e)–5(g)). A pretreatment with RRE, especially at 5 ng/ml concentration, was able to reduce the Dexa-induced cytosolic, mitochondrial, and mitochondrial superoxide ROS levels by up to 16.9%, 22.0%, and 22.1%, respectively (Figures 5(a)–5(c)). The most effective concentrations of the extract that significantly decreased ROS levels to those of the control condition were 5 and 10 ng/ml for cytosolic ROS (Figure 5(a)), 5 ng/ml for mitochondrial ROS (Figure 5(b)), and 10 ng/ml for mitochondrial superoxide anion (Figure 5(c)). Pretreatment with the same RRE concentrations was able to rescue the decrease in cellular metabolic activity (an indicator of cell viability) caused by 400 *μ*M Dexa (Figure 5(d)). Namely, a pretreatment with 1, 5, and 10 ng/ml of the RRE rescued the cell viability by up to 12.2%, almost a complete rescue. Of note, these effects are not unique to the SH-SY5Y cells. Indeed, a similar effect was observed in the HT22 cells in which Dexa 5 *μ*M treatment caused an elevation of the same type of ROS (Suppl. Figures 1(a)–1(c)). A pretreatment with RRE, especially the 5 ng/ml and 10 ng/ml concentrations, significantly reduced cytosolic ROS, mitochondrial ROS, and mitochondrial superoxide anion. In line with data obtained in SH-SY5Y cells, Dexa 100 *μ*M caused a decrease in cellular metabolic activity compared to the control in HT22 cells (Suppl. Figure 1(d)). Treatment with 5 and 10 ng/ml of the RRE rescued cell metabolic activity up to 16.1%.

Strikingly, the protective effects of RRE against Dexa-induced oxidative damages were also observed with a curative treatment (Figures 4(e)–4(h)). Indeed, in the presence of 100 *μ*M Dexa, RRE 5 ng/ml decreased the cytosolic ROS to the level of the untreated SH-SY5Y cells (Figure 5(e)). Moreover, RRE normalized mitochondrial ROS and mitochondrial superoxide anion levels in the presence of Dexa, with 5 ng/ml being the most effective concentrations decreasing mitochondrial ROS by 20.5% and mitochondrial superoxide anions by 20.3% compared to cells treated with Dexa alone (Figures 5(f) and 5(g)). In line, RRE 5 ng/ml normalized the cellular metabolic activity of Dexa-treated cells to the level of the control cells (Figure 5(h)).

Taken together, these data showed that RRE rescued cell metabolic activity and decreased ROS levels under corticosteroid stress. Again, the effects of RRE presented a U-shape (for ROS) and inverted U-shape (for cell metabolic activity), with 5 and 10 ng/ml being the two most efficient extract concentrations.

### 3.6. RRE Increases Neurite Outgrowth and BDNF Expression under Stress Condition

In a next step, we assessed the capacity of RRE in promoting neurite outgrowth in SH-SY5Y cells under stress condition and subsequent immunostaining and microscopy analysis (Figure 6). The most promising RRE concentration from the previous experiments (5 ng/ml) was used as curative treatment to test its effect on neurite outgrowth (Figure 6(a)). As for the ROS experiments, Dexa at 100 *μ*M was used to induce stress and caused a decrease of 52.4% in neurite count, a decrease of 41.1% in total neurite length, a decrease of 43.4% in the number of attachment points, and a decrease of 47.6% in the number of endpoints, when compared to the untreated control cells (Figures 6(b)–6(e)). RRE 5 ng/ml was able to counteract the effects of Dexa by increasing the neurite count (Figure 6(b)), total neurite length (Figure 6(c)), number of attachment points (Figure 5(d)), and number of endpoints (Figure 6(e)) by 20.2%, 22.8%, 23.2%, and 21.2%, respectively, compared to the cells treated with Dexa alone.

Because RRE increases BDNF expression in basal condition, we next examined whether this effect is also observed in stress condition. Dexa induced a decrease of about 20% of BDNF mRNA level, while a curative treatment with RRE restored BDNF expression to the level of the untreated control cells (Figure 6(f)). Cellular actions of BDNF are mediated through two main receptors: tyrosine receptor kinase B (TrkB) and p75 neurotrophin receptor (p75NTR). Therefore, we next assessed whether RRE modulates TrkB and p75NTR expression under normal condition or under Dexa-induced stress. Although RRE or Dexa alone tended to increase TrkB, the difference with the control cells was not significant (Figure 6(b)). However, a 47.5% increase in TrkB expression was observed after RRE treatment under stress condition, when compared to the control condition. Strikingly, RRE strongly decreased p75NTR expression (-87% compared to untreated cells), while Dexa upregulated its expression (+72% compared to the control). A combined treatment of RRE and Dexa decreased of about 25% p75NTR expression compared to cells treated with Dexa alone (Figure 6(b)). These data demonstrate that RRE 5 ng/ml reduces the damages caused by Dexa, by promoting neurite growth and connectivity and modulating BDNF, TrkB, and p75NTR expression.

## 4. Discussion

In this study, we hypothesized that WS®1375 extract of the adaptogenic plant *Rhodiola rosea* can reduce the detrimental effects of glucocorticoid-induced stress. The basal effect of RRE was examined at a concentration range of 1-100 ng/ml on two cell lines: the human neuroblastoma cells SH-SY5Y which is a known and well-characterized neuronal model and the murine hippocampal cell line HT22. The latter cell line was selected in order to confirm our results in cells generated from a brain structure that is at the forefront of the impact of glucocorticoid stress as the hippocampus highly expresses GRs [43]. Dexamethasone, a synthetic glucocorticoid mimicking the effect of the endogenous stress hormone cortisol, was used to simulate a glucocorticoid-induced stress. Two treatment conditions were tested on SH-SY5Y cells: a preventive treatment, in which cells were first treated with RRE for 24 h and then treated with Dexa for another 24 h, and a curative treatment, in which cells were first stressed with Dexa for 3 h and additionally treated with RRE for 24 h. The rational underlying this approach in everyday life is that RRE might be taken in prevision of a stressful event (e.g., examination session and upcoming conflict) to reduce the effect of stress, or during a stressful period to counteract the effect of stress.

Our key results were that (i) RRE increased ATP levels and cell metabolic activity in an inverted U-shaped dose response curve, in line with the adaptogenic nature of this plant extract; (ii) RRE pretreatment (preventive) and posttreatment (curative) reduced Dexa-induced increase of ROS and decrease of cell metabolic activity; and (iii) RRE increased neurite outgrowth and BDNF expression, both in healthy and stressed conditions.  Figure 7 summarizes these key results.

Mitochondria are the main generators of ROS and are directly affected by their overproduction. At the same time, neurons are highly dependent on mitochondria for their function and survival as they demand high amounts of energy, while they are more vulnerable to oxidative stress [44–46]. In our study, Dexa significantly increased the levels of mitochondrial ROS, cytosolic ROS, and mitochondrial superoxide anion in both cell lines. Moreover, Dexa induced a decrease in cell metabolic activity in SH-SY5Y and HT22 cells that might be related to the Dexa-induced increase in ROS production. Both preventive and curative RRE treatment rescued the cell survival and normalized ROS levels after Dexa-induced stress, with the 5 ng/ml concentration being the most effective. In line with these data, glucocorticoids such as cortisol have been shown to increase ROS production leading to an oxidative stress state [27, 47, 48] with increased oxidation markers such as 8-hydroxyguanosine (8-oxoG) and 8-iso-prostaglandin F2*α* (IsoP) as demonstrated in the saliva of chronically stressed women [27]. Consistently, it has been shown that anongenomic glucocorticoid receptor-mediated pathway can also lead to increased ROS production with concomitant activation of the ERK/CREB/PGC1-*α* signaling as a stress compensation mechanism in the rainbow trout [47].

In both treatment conditions (preventive and curative), the protective effect of RRE on the Dexa-induced increase of ROS displays U-shaped dose response curves as illustrated in Figure 5. Accordingly, inverted U-shaped dose response curves showing the effects of RRE on the impaired cell viability induced by Dexa have been observed (see Figure 5, D and H). Importantly, these data clearly indicate that RRE decreases ROS levels and increases cell viability event when stress is already initiated. Those biphasic response curves are usually characteristic for botanicals, especially plant adaptogens [17, 49–51]. Typically, low doses of an adaptogen induce a dose-dependent increase in biological response until a maximum response is reached. Higher doses induce a gradual decrease in the response until it might even reach a nonobservable effect level, a phenomenon also called hormesis [49]. Thus, a biphasic response curve could reflect activation of the «adaptive cellular stress response». Our findings are in line with RRE-induced U-shaped dose response curves reported by others in human osteosarcoma-derived 143B, human diploid fibroblast IMR-90, and human neuroblastoma IMR-32 cells under paraquat, H_2_O_2_, and UV stress [17], as well as in mice [52]. U-shaped response curves have been also shown on the lifespan of *C. elegans* after treatment with the adaptogens *Eleutherococcus senticosus* and *Rhodiola rosea*. Consistently, our findings confirm that the herbal RRE WS®1375 exhibits the typical features of an adaptogen with regard to the modulation of adaptive homeostasis and stress response.

Furthermore, our data are in line with existing literature supporting the antioxidant effect of RRE and especially of its compound salidroside [21, 53–58]. Indeed, an ethanolic RRE containing high concentrations of phenolic compounds, particularly salidroside, showed a strong antioxidant activity in the 1,1-diphenyl-2-picrylhydrazyl scavenging capacity assay (DPPH), in the 2,2'-azino-bis(3-ethylbenzothiazoline-6-sulphonic acid) scavenging capacity assay (ABTS), and in the ferric reducing antioxidant power assay (FRAP) [55]. In line, a very recent study showed that *Rhodiola rosea* rhizomes, especially the two bioactive compounds salidroside and tyrosol, showed free radical scavenging activity when assessed in the ABTS and DPPH assays, while it also normalized dihydrochloride-induced increase of ROS in PC12 cells [59]. Additionally, salidroside protected PC12 cells from H_2_O_2_-induced apoptosis through inactivation of the caspase cascade and through prevention of cytochrome c release [53]. Both, salidroside and tyrosol, abolished the H_2_O_2_-induced oxidative damage in rat cortical neurons by decreasing the expression of Bax (a proapoptotic protein) with tyrosol being more effective possibly due to its position of the glycosyl group [56].

RRE pretreatment protected human cortical cells (HCN 1-A) against H_2_O_2_- and glutamate-induced cell apoptosis by normalizing the stress-induced increase in intracellular calcium concentration [18]. Salidroside exerted the same effects but in a lower extent than the extract indicating that the neuroprotective effect of RRE is a result of synergistic effect of its compounds. An ethyl acetate RRE fraction (50 *μ*g/mL) demonstrated the highest cell viability values during methylglyoxal-induced apoptosis in neuro-2A (N2A) cells, while salidroside (50 *μ*M 24 h) exhibited the strongest neuroprotective activity among the tested compounds of the ethyl acetate fraction [60]. Moreover, in SH-SY5Y cells, salidroside was able to rescue the H_2_O_2_-induced cell death by increasing antioxidant enzymes such as thioredoxin, heme oxygenase-1, and peroxiredoxin-I, by downregulating the proapoptotic gene Bax, as well as by upregulating the antiapoptotic gene Bcl-2, mechanisms that might also be involved in the observed effects of the RRE WS®1375 [21]. Interestingly, salidroside showed also neuroprotective effects in SH-SY5Y cells expressing the amyloid precursor protein (APP), a cellular model of Alzheimer's disease (AD) [61]. Indeed, salidroside was able to inhibit the hypoxia-induced amyloid-*β* generation by decreasing *β*-secretase activity and decreasing BACE1 (beta-site APP cleaving enzyme 1) expression.

Most of cellular ROS are produced by mitochondria as by-products of OXPHOS which takes place at the electron transport chain (ETC) on the inner mitochondrial membrane. ROS are mainly generated by complexes I and III of the ETC when leaking electrons that are provided by NADH or FADH_2_ react with oxygen [38, 62]. Since our findings indicated that RRE neutralized mitochondrial and cellular ROS, we aimed to examine the potential effect of the extract on increasing mitochondrial functions such as ATP production and metabolic activity. As mentioned before, mitochondria are at the epicenter of neuronal health and survival mainly because they are the principal energy producers and suppliers (in the form of ATP). The main mechanism leading to the production of ATP is OXPHOS that takes place in the ETC of mitochondria [44, 46]. RRE concentrations (1-100 ng/ml) had a positive effect on both ATP production and metabolic activity after 24-h treatment of the two cells lines. The RRE concentrations that increased the most the ATP production and the metabolic activity were the 5 and 10 ng/ml. Again, we could confirm that the effects of RRE follow the typical biphasic dose response curves of adaptogens in two different neuronalcell lines (see Figure 2).

Apart from one study conducted two decades ago showing that RRE increased ATP levels in mitochondria of skeletal muscles in rats, there are no further specific studies evaluating the effect of the RRE or its compounds on bioenergetics [63]. Another study indicated the beneficial effect of the extract of another *Rhodiola* species, that of *Rhodiola crenulata*, which increased the ATP production and cell viability as well as reduced the loss of neurons in the hippocampus of rats with hypobaric hypoxia [64]. However, different *Rhodiola* species contain different bioactive compounds. For example, rosavin is a characteristic marker of RRE and is not present in many other *Rhodiola* species such as *Rhodiola crenulata* [65, 66]. Therefore, it can be speculated that rosavin does not contribute to the ATP-increasing effect of RRE in neuronal cells. Of note, salidroside (1 *μ*mol/l) showed protective effects against mitochondrial dysfunction induced by oxygen-glucose deprivation (OGD, mimicking the effects of ischemia in vitro) in HT22 cells [67]. Namely, cell viability was restored after salidroside treatment, together with a decrease in mitochondria fragmentation and inhibition of excessive mitophagy caused by OGD. This indicates that the effect we observed on bioenergetics might preferentially be linked to the presence of salidroside in our RRE WS®1375.

Healthier mitochondria lead to healthier neurons which can fulfill their functions most efficiently. One of the main functions of neurons is to form interconnections with nearby neurons, namely, synapses. The ability to form synapses in response to neuronal needs is called synaptic plasticity, and it represents the cellular mechanisms of learning and memory [68]. Mitochondria are playing a major role in synaptic plasticity as the main energy suppliers and calcium concentration regulators [68]. Since the RRE had a positive effect on mitochondrial functions, we further examined its effect on neurite outgrowth. Neurite outgrowth is the growth and elongation of neuronal axons and dendrites that subsequently leads to the formation of synapses and synaptic plasticity [69]. A commonly used model to study neurite outgrowth is differentiated SH-SY5Y cells [39]. Upon analysis and quantification of neurite outgrowth parameters, we showed that RRE caused a significant increase in the number of neurites, in the total neurite length, in the attachment points of neurons and in the number of endpoints of neurons.

Since RRE promoted neurite outgrowth, we examined whether the growth factor BDNF was involved in this process. Indeed, BDNF belongs to the protein family of neurotrophins, which are mediating synaptic processes. BDNF is the main neurotrophin that regulates synaptic plasticity and neurite outgrowth as it is highly expressed in many brain regions including the hippocampus and cortex. Its expression plays a critical role in learning and memory [70, 71]. Treatment with RRE caused a fast-upregulating effect on the BDNF mRNA expression peaking at 3 h. Our findings are in line with previous research showing that salidroside, one of the lead compounds in RRE, has an upregulating effect on mRNA BDNF levels [22]. Our study is the first evaluating the effect of the whole extract on mRNA BDNF levels. Of note, increased BDNF mRNA expression does not necessarily lead to increased BDNF protein levels because the mRNA could possibly not be translated into the respective protein that is necessary for the induction of neurite outgrowth and synaptic plasticity. BDNF is synthetized as a preform that includes a prosegment and the mature BDNF. The prosegment is removed by proteases and the secreted mature BDNF binds to its receptor TrkB inducing long-term potentiation, while the pro-BDNF binds to the receptor p75 causing long-term depression [71]. The production of mature BDNF is a posttranslational process. Therefore, we further evaluated the effect of RRE on the level of mature BDNF protein. We observed an increase in the level of mature BDNF level after a few hours of treatment. In line with this, several studies demonstrated that the BDNF system is a fast-reacting one. Thus, mRNA expression started already to increase after 15 min of induced middle cerebral artery occlusion peaking at 2 h after reperfusion in cortical neurons from the rat brain [40] and was accompanied by elevated levels of BDNF protein peaking at 2 h [72] of reperfusion (following 2 h of middle cerebral artery occlusion). Consistent with our findings, intrahippocampal infusion of spermidine, a natural polyamine exhibiting antioxidant properties, increased the mature BDNF protein level in a similar fast time frame as did RRE, namely, after 3 h of treatment [41]. We can speculate that the effects of RRE on the BDNF system are related to its beneficial effect on neurite outgrowth and network connectivity. Interestingly, salidroside, rosavin, and other commercial RRE potentiated electric stimulation of an intrahippocampal electric circuit resulting in higher responses of the pyramidal cells in isolated hippocampus slices [73]. One can speculate that the effects of different RRE and related bioactive compounds (salidroside and rosavin) on neuronal activity may also be linked to an increase in bioenergetics. The exact mechanisms remain to be determined.

Most importantly, we showed that RRE curative treatment increases neurite outgrowth and BDNF expression under Dexa-induced stress. Indeed, Dexa drastically reduced neurite count and length as well as neuronal connectivity in differentiated SH-SY5Y cells and induced a significant decrease of BDNF mRNA level (Figure 6). These data are in line with previous studies showing the deleterious effects of glucocorticoid-related stress on neuroplasticity (reviewed in [35]). To our knowledge, we are the first to show that RRE rescues the deleterious effects of Dexa by increasing all the above-mentioned parameters. We can hypothesize that the effects observed on neurite outgrowth can either be due to the scavenging properties of RRE, which possibly increase neuronal health and neuroplasticity, or be due to the modulatory effects of RRE on the BDNF pathway (Figure 7). Indeed, our data indicate that a treatment with Dexa decreases BDNF mRNA expression, does not alter TrkB mRNA expression, and increases p75NTR mRNA expression. These data are in line with previous studies showing a downregulation of BDNF mRNA, with no effect on TrkB mRNA level, as well as an increase in p75NTR immunoreactivity in the hippocampus of Dexa-treated animals [74, 75]. While mature BDNF binds TrkB with high affinity and promotes cell survival, the BDNF precursor, called proBDNF, binds p75NTR with high affinity leading to apoptosis [76]. Therefore, our data suggest that, in our model, Dexa decreases cell viability and neuroplasticity by decreasing BDNF mRNA level and favors the proapoptotic p75NTR pathway by increasing p75NTR expression. Strikingly, a posttreatment with RRE normalized BDNF mRNA level, increased TrkB expression, and downregulated p75NTR mRNA. These findings indicate that RRE may counteract the effects of Dexa by increasing BDNF levels and inhibiting the p75NTR pathway. Additional experiments are now needed to dissect in more details the underlying mechanisms.

On the basis of our results, we can suggest that RRE constitutes an adaptogenic candidate with the potential to combat stress-induced impairment by acting either (i) directly on mitochondria, resulting in enhanced synaptic transmission, or (ii) by possibly exerting its properties indirectly by increasing BDNF levels which then in turn enhances mitochondrial functions and induces neurite outgrowth (Figure 7).

## 5. Conclusion

Overall, in this study, we showed that the RRE WS®1375 neutralizes the harmful effect of corticosteroid stress, regulates neuronal ROS levels, and improves neuronal survival in stressful situations. RRE WS®1375 exhibited a biphasic U-shaped dose response curves that are typical for adaptogens constituting the activation of the «adaptive cellular stress response». In addition, we demonstrated that the RRE increased mitochondrial bioenergetics as well as promoted neurite outgrowth in neuronal cells under normal and stressed conditions. The mechanism underlying the promotion of neurite outgrowth might be the BDNF pathway as RRE upregulated both the BDNF mRNA and the mature BDNF protein levels. Although there are some studies demonstrating the antioxidant and neuroprotective effect of salidroside, one of the postulated lead compounds of RRE, there are very few studies examining the effect of a whole extract on these parameters, and no studies (until now) had investigated the effects of RRE in glucocorticoid-mediated stress condition. More research is needed to characterize the effect of different compounds of RRE such as rosavin, rosarin, and tyrosol. This is particularly interesting since the efficacy of the RRE could be a result of antagonistic, synergistic, or allosteric effects of its constituents. Finally, our findings indicate that RRE could constitute a candidate for combatting stress-induced ailments and stress-associated mental disorders with the involvement of oxidative stress and could potentially lead to the establishment of a condition-specific supplement.

## Figures and Tables

**Figure 1:** HPLC-UV fingerprint of WS®1375 detected at 275 nm. The quantified analytes are marked. The single WS®1375 batch used for the present study contained 1.04% rosarin, 2.63% rosavin, 1.04% rosin (all assessed as rosavins), and 1.16% salidroside (assessed as p-tyrosol).

**Figure 2:** Effect of RRE on ATP production and cell viability. (a) RRE at 1-100 ng/ml significantly increased the ATP production in SH-SY5Y cells after 24 h of treatment. (b) RRE at 5 and 10 ng/ml significantly increased the cell metabolic activity in SH-SY5Y cells after 24 h. (c) Pearson correlation between ATP production and metabolic activity revealed a significant positive linear correlation after 24 h of treatment (*R*^2^ = 0.9007, *p* = 0.0137) with the most effective RRE concentrations being 5 and 10 ng/ml. (d) RRE at 1-100 ng/ml significantly increased the ATP production in HT22 cells after 24 h of treatment. (e) RRE at 5 ng/ml significantly increased the cell metabolic activity in HT22 cells after 24 h. (f) A significant positive linear correlation was found between the ATP production and the metabolic activity in HT22 cells after 24 h of treatment (*R*^2^ = 0.8616, *p* = 0.0228). The square symbols are used for SH-SY5Y cells (c), and the circle symbols are used for HT22 cells (f). Values represent the mean ± SEM of three independent experiments. For statistics, one-way ANOVA and post hoc Dunnett's multiple comparison test versus untreated (CTRL) were used (a, b, d, e). The adequacy of fits was estimated by the *R*-squared value (>0.9) using Pearson correlation and linear regression analysis (c, f). Values represent the mean of the survival in ordinate and the mean of ATP concentration in abscissa. ∗*p* < 0.05, ∗∗*p* < 0.01, and ∗∗∗*p* < 0.001.

**Figure 3:** Neurite outgrowth in differentiated SH-SY5Y cells. (a) RRE at 5 and 10 ng/ml increased the neurite outgrowth of SH-SY5Y cells after 3 days of treatment. Pictures were taken using a digital microscope of a multimode plate reader (×20). Immunostaining was performed with *β*III-tubulin/Alexa fluor-488 for the soma and neurites. The nucleus was stained using DAPI. Pictures display neurite extension between the cells (upper panels). Neurite outgrowth parameters such as the attachment points (middle panels) and the endpoint numbers (lower panels), after NGF (50 ng/ml), BDNF (50 ng/ml), or RRE at 5 and 10 ng/ml treatment are illustrated (blue and gray: soma; red: neurites; green points: attachment points; yellow points: endpoints). (b–e) Quantification of neurite outgrowth was performed using NeurophologyJ. At 5 and 10 ng/ml RRE significantly increased: (b) number of neurites (neurite count), (c) neurite length, (d) number of attachment points, and (e) number of endpoints. The effect of RRE was similar to that of the positive controls NGF and BDNF when compared to the untreated cells (CTRL). Values represent the mean ± SEM of three independent experiments. For statistics, one way ANOVA and post hoc Dunnett's multiple comparison test versus untreated (CTRL) was used, ∗∗∗*p* < 0.001.

**Figure 4:** BDNF mRNA and mature BDNF protein levels in SH-Y5Y cells. (a) The effect of 5 ng/m RRE peaked after 3 h of treatment with a significant increase in the BDNF mRNA expression. Data are normalized to 1 (corresponding control condition) and presented as mean ± SEM of three independent experiments. (b) Treatment with RRE at 5 ng/ml had as well an upregulating effect on the protein level of mature BDNF exhibiting a significant increase at 4 h. Data are normalized to 1 (corresponding control condition) and presented as mean ± SEM of three independent experiments. Values represent the mean ± SEM of three independent experiments. For statistics, unpaired Student *t* test versus the corresponding untreated (CTRL) of each time point was used, ∗*p* < 0.05, ∗∗*p* < 0.01, ∗∗∗*p* < 0.001, and ∗∗∗∗*p* < 0.0001.

**Figure 5:** Effect of RRE pre-treatement (preventive) and posttreatment (curative) on ROS levels and cell metabolic activity in SH-SY5Y cells under dexamethasone-induced stress. (a) Pretreatment with RRE at 5 and 10 ng/ml reduced significantly the Dexa-induced increase in cytosolic ROS. (b) Dexa-induced increase in mitochondrial ROS was significantly reduced by a pretreatment with RRE 5 ng/ml. (c) Pretreatment with RRE at 10 ng/ml significantly reduced the Dexa-induced increase in mitochondrial superoxide anion levels. (d) A pretreatment with the RRE concentrations 1-10 ng/ml significantly rescued cell metabolic activity of dexa-treated SH-SY5Y cells. (e) Treatment with RRE at 5 ng/ml (curative) reduced significantly the Dexa-induced increase in cytosolic ROS. (f) Dexa-induced increase in mitochondrial ROS was significantly reduced by a treatment with RRE 1-100 ng/ml. (g) Treatment with RRE at 5 and 10 ng/ml significantly reduced the Dexa-induced increase in mitochondrial superoxide anion levels. (h) Treatment with the RRE concentration 5 ng/ml significantly rescued cell metabolic activity of dexa-treated SH-SY5Y cells. Values represent the mean ± SEM of three independent experiments and were normalized on the untreated group (=100%). One-way ANOVA and post hoc Dunnett's multiple comparison test versus Dexa were used. ∗*p* < 0.05, ∗∗*p* < 0.01, and ∗∗∗*p* < 0.001.

**Figure 6:** Neurite outgrowth and BDNF pathway in SH-SY5Y cells under Dexa-induced stress. (a) RRE WS®1375 at 5 ng/ml reduced the dexamethasone-induced damage on neurite outgrowth in SH-SY5Y cells. Pictures were taken using a digital microscope of a multimode plate reader (×20). Immunostaining was performed with *β*III-tubulin/Alexa Fluor-488 for the soma and neurites. The nucleus was stained using DAPI. Pictures display neurite extension between the cells (upper panels). Neurite outgrowth parameters such as the attachment points (middle panels) and the endpoint numbers (lower panels) are illustrated in the untreated cells (CTRL), cells treated with Dexa 100 *μ*M, and cells treated with Dexa 100 *μ*M and then with WS®1375 at 5 ng/ml (blue and gray: soma; red: neurites; green points: attachment points; and yellow points: endpoints). (b–e) Dexa decreased all four parameters of neurite outgrowth compared to control (normalized to 100%; dotted line). WS®1375 was able to ameliorate this decrease. Quantification was performed using NeurophologyJ. At 5 ng/ml, WS®1375 significantly increased: (b) number of neurites (neurite count), (c) neurite length, (d) number of attachment points, and (e) number of endpoints under Dexa stress. (f) RRE 5 ng/ml modulate the mRNA level of BDNF TrkB and p75NTR under Dexa stress. Values represent the mean ± SEM of two independent experiments. A total of 15-21 pictures per condition were taken and analyzed. For statistics, one-way ANOVA and post hoc Dunnett's multiple comparison test versus corresponding dexamethasone (dexa) concentration were used. ∗*p* < 0.05, ∗∗*p* < 0.01, and ∗∗∗*p* < 0.001.

**Figure 7:** Possible pathway involved in protective effects of RRE against glucocorticoid-induced stress. Chronic stress is known to disturb the BDNF pathway, leading to a decreased synaptic plasticity and neurite outgrowth. Data obtained in the present study confirms the effects of dexamethasone (Dexa-)-induced stress on neuronal cells (see red arrows on the scheme). RRE seems to counteract the effects of Dexa by increasing BDNF level and TrkB-dependent signaling pathway leading to an increase in cell survival and neuroplasticity (see green arrows on the scheme). In parallel, RRE normalizes bioenergetic impairments induced by Dexa, by increasing ATP levels and decreasing mitochondrial ROS production. Of note, as BDNF was also shown to modulate mitochondrial bioenergetic activity, RRE may also act indirectly on mitochondria by increasing BDNF levels. This figure was created with http://BioRender.com. ATP: adenosine triphosphate; BDNF: brain-derived neurotrophic factor; p75NTR: p75 neurotrophin receptor; ROS: reactive oxygen species; RRE: Rhodiola rosea extract (here: WS®1375); TrkB: tyrosine receptor kinase B.

## Data Availability

Data are available on request after contacting Professor Dr. Anne Eckert (anne.eckert@upk.ch).

## Abbreviations

ABTS: 2 : 2'-Azino-bis(3-ethylbenzothiazoline-6-sulphonic acid) scavenging capacity assay
ACTH: Adrenocorticotropic hormone
ATP: Adenosine triphosphate
Bax: Bcl-2-associated X protein
Bcl-2: B-cell lymphoma 2 protein
BDNF: Brain-derived neurotrophic factor
BSA: Bovine serum albumin
cDNA: Complementary DNA
CXR: Carboxy-X-rhodamine reference dye
DAPI: 4′,6-Diamidino-2-phenylindol
DCF: 2',7'-dichlorodihydrofluorescein diacetate
Dexa: Dexamethasone
DHR: Dihydrorhodamine 123
DMEM: Dulbecco's modified eagle medium
DMSO: Dimethyl sulfoxide
DNA: Deoxyribonucleic acid
DPPH: 1,1-Diphenyl-2-picrylhydrazyl scavenging capacity assay
ELISA: Enzyme-linked immunosorbent assay.
ERK/CREB/PGC1-*α*: Extracellular signal-regulated kinase/cAMP Response Ele-ment-binding Protein/Peroxisome proliferator-activated receptor-gamma coactiva-tor-1alpha.
ETC: Electron transport chain
FADH2: Reduced form of flavin adenine dinucleotide (FAD)
FCS: Fetal calf serum
FRAP: Ferric reducing antioxidant power assay
GAPDH: Glyceraldehyde 3-phosphate dehydrogenase gene
HBSS: Hanks' balanced salt solution
HPA: Hypothalamic–pituitary–adrenal axis
HT22: Immortalized mouse hippocampal cell line
IsoP: 8-iso-prostaglandin F2*α*
MitoSOX: Mitochondrial superoxide anion dye
mRNA: Messenger RNA
MTT: 3-(4,5-dimethylthyazol-2-yl)-2,5-diphenyl-tetrazolium bromide
NADH: Reduced form of nicotinamide adenine dinucleotide
NGF: Nerve growth factor
OXPHOS: Oxidative phosphorylation
p75NTR: p75 neurotrophin receptor
PBS: Phosphate-buffered saline
PC12: Phaeochromocytoma cells from rat adrenal gland
PCR: Polymerase chain reaction
qPCR: Quantitative polymerase chain reaction
RA: Retinoic acid
RRE: *Rhodiola rosea* extract
RNA: Ribonucleic acid
ROS: Reactive oxygen species
S.E.M.: Standard error of the mean
SH-SY5Y: Human neuroblastoma cell line
TrkB: Tyrosine receptor kinase B
WS®1375: Specific *Rhodiola rosea* extract (Dr. Willmar Schwabe GmbH & co KG, Karlsruhe, Germany) used in this study
8-oxoG: 8-hydroxyguanosine

## Supplementary Materials

Supplementary Materials Supplementary Figure 1. Effect of RRE on ROS levels and cell metabolic activity in HT22 cells under dexamethasone-induced stress. (a) RRE at 5 ng/ml significantly decreased the Dexa-induced cytosolic ROS. (b) Dexa-induced increase in mitochondrial ROS was significantly reduced by RRE. (c) RRE at 1-10 ng/ml significantly reduced the Dexa-induced increase in mitochondrial superoxide anion levels. (d) The cell viability was decreased in Dexa-treated HT22 cells. The RRE concentrations 5 and 10 ng/ml prevented this decrease. Values represent the mean ± SEM of three independent experiments and were normalized on the untreated group (=100%). One-way ANOVA and post hoc Dunnett's multiple comparison test versus Dexa were used. ∗*p* < 0.05, ∗∗*p* < 0.01, and ∗∗∗*p* < 0.001. Supplementary Table 1: Effect of RRE on cell viability in SH-SY5Y cells (prescreening) Supplementary Table 2: Effect of RRE on cell viability in HT22 cells (prescreening).
